The article "Study on BCVA, CMT, CME, Curative Effect, and Prognostic Value of DR Sufferers Based on Surgical Therapy Combined with VEGF Therapy at Different Times" was retracted in 2023. Reasons: signs of a paper mill; suspected computer-generated content; unreliable results or conclusions; concerns about the data.

# Study on BCVA, CMT, CME, Curative Effect, and Prognostic Value of DR Sufferers Based on Surgical Therapy Combined with VEGF Therapy at Different Times

**DOI:** 10.1155/2022/1415659

**Published:** 2022-08-11

**Authors:** Jian Wang

**Affiliations:** Shaoxing Shangyu People's Hospital, Shaoxing 312300, China

## Abstract

In order to explore the efficacy and prognostic value of best corrected visual acuity (BCVA), central macular retinal thickness (CMT), and cystoid macular edema (CME) in diabetic retinopathy (DR) sufferers based on surgical therapy combined with vascular endothelial growth factor (VEGF) therapy at different times, a total of 170 cases of DR sufferers who visited our hospital from March 2019 to March 2021 are analyzed. All patients are randomly divided into control group and study group, with 85 cases and 85 eyes in each group. In addition, the contrast set received 2 therapies for 1.5 months/time, and the study set received 3 therapies for 1 month/time. The experimental results show that the BCVA of the two sets is notoriously enhanced. Besides, CMT and CME in the study set decrease more than those in the contrast set, and the blood vessel density of retinal capillaries in the contrast set and the examination set is notoriously enhanced. For DR sufferers, 1 month/time of anti-VEGF therapy can effectively enhance the sufferers' visual acuity, CMT and CME. It is suggested that the clinical application of 1 month/time of anti-VEGF to DR sufferers can enhance the clinical therapeutic effect of sufferers and reduce the prognosis and recurrence.

## 1. Introduction

Among diabetic microangiopathy, diabetic retinopathy (DR) is one of the more serious complications. The prevalence of DR in diabetic sufferers over 40 years old is as high as 34.6%. DR can be clinically divided into nonproliferative and proliferative stages according to the presence or absence of retinal neovascularization [1]. Among them, proliferative diabetic retinopathy (PDR) is seriously harmful, and its retinal neovascularization is prone to hemorrhage, which will further lead to vitreous hemorrhage. In addition, the neovascularization may also fibrosis and shrink, forming an epiretinal membrane and causing traction retinal detachment, which seriously affects vision [2, 3]. Generally speaking, diabetes retinopathy begins with slight degeneration of retinal microvessels [4]. Once this condition occurs, it will develop into a more serious condition that endangers vision. In proliferative retinopathy, abnormal new blood vessels grow on the surface of the retina. These fragile new blood vessels are very easy to rupture, and blood will flow to the middle part of the eye and hinder vision. This neovascularization is also very easy to atrophy, and the scar tissue formed by its atrophy may also form around the retina, eventually leading to retinal detachment. In addition, the fluid in the blood will continue to leak from retinal vessels, resulting in macular edema [5]. The macula is part of the retina and is responsible for providing sharp and clear vision when reading and driving. When an important part of the macula swells due to too much liquid, the vision will become very blurred, making it difficult to play or lose its function [6]. Macular edema cannot affect vision until it develops to a certain time, like microangiopathy [7]. It can appear at any stage of diabetes and seriously affects vision from the beginning. Vascular Endothelial Growth Factor (VEGF) is an important factor for retinal neovascularization in PDR. Therefore, anti-VEGF therapy is usually used in the clinical treatment of retinopathy [8]. Due to the lack of research on the relevant examination of the best treatment time, this study will select DR patients as the research object to analyze the efficacy and prognostic value of anti-VEGF treatment at different times.

The article "Study on BCVA, CMT, CME, Curative Effect, and Prognostic Value of DR Sufferers Based on Surgical Therapy Combined with VEGF Therapy at Different Times" was retracted in 2023. Reasons: signs of a paper mill; suspected computer-generated content; unreliable results or conclusions; concerns about the data.

The rest of this paper is organized as follows: Section 2 presents the related work. The examination objects and methods are presented in Section 3.  Section 4 presents the comparative results.  Section 5 concludes the paper.

## 2. Related Work

The pathological changes of DR are ocular nerve and blood vessel microcirculation disorders, resulting in abnormal eye nutrition and damage to visual function. VEGF is the most critical factor in causing new blood vessel growth and microcirculation abnormalities, especially in the preclinical stage of DR to proliferation [9]. Conbercept can target and inhibit human Vascular Endothelial Growth Factor A (VEGF-A), and the application of Conbercept in the therapy of Diabetic Macular Edema (DME) is effective. Intravitreal injection of Conbercept is known as an invasive therapy method. Currently, intravitreal injection of widely used anti-VEGF drugs also can cause serious complications, such as endophthalmitis. Especially when anti-VEGF drugs are injected repeatedly, the risk of endophthalmitis is further increased, and intravitreal hemorrhage and retinal detachment may also be caused. Moreover, repeated injections will lead to higher treatment costs [10]. Therefore, it is necessary to explore the clinical effect and safety of Conbercept in the therapy of DME. Observing the number of therapies or the dose and frequency of injections is of great significance for the diagnosis and therapy of DR sufferers.

Anti-VEGF therapy has a certain effect on DR, which is characterized by the development of ischemic retinopathy. Studies have found that after intravitreal injection of anti-VEGF drugs in DR, the retinal nonperfusion area is reduced and the ischemia condition is enhanced [11]. Some studies found that the severity of retinopathy in the Conbercept set decreased and the progression is delayed. From a practical point of view, oxidative stress, hypoxia, and inflammatory responses can induce increased VEGF expression [12]. The increase in VEGF level plays an important role in promoting the occurrence and development of new blood vessels. The concentration of VEGF in the vitreous humor of PDR sufferers is notoriously increased. Anti-VEGF therapy can effectively inhibit VEGF and regress new blood vessels [13]. At the same time, in sufferers with DME, anti-VEGF therapy can also reduce edema and enhance visual acuity. Because intravitreal injection of anti-VEGF drugs is an invasive operation, especially when endophthalmitis is caused, it often leads to a very high risk of blindness in sufferers, so it should be strictly sterile. Operation and local administration of antibiotics may be necessary [14].

The article "Study on BCVA, CMT, CME, Curative Effect, and Prognostic Value of DR Sufferers Based on Surgical Therapy Combined with VEGF Therapy at Different Times" was retracted in 2023. Reasons: signs of a paper mill; suspected computer-generated content; unreliable results or conclusions; concerns about the data.

The avascular area of the Foveal Avascular Zone (FAZ) is a key index for the detection of retinal diseases. FAZ is essential for maintaining fine vision. Many scholars believe that the loss of central vision in DR may be due not only to macular edema itself but also to changes in FAZ [15, 16]. Intravitreal injection of Conbercept in the therapy of DR can enhance the blood supply of the deep capillary plexus in the fovea and parafoveal retina, and reduce the number of microvascular tumors, while the blood supply of the superficial capillary plexus and the number of microvascular tumors are not obvious. The changes suggest that Conbercept injection can enhance the blood circulation and distribution in the central fovea and parafoveal retina, and the increase in the number of injections can further enhance its clinical effect [17]. In the decomposition of the vitreous humor of DR sufferers, it is found that the content of VEGF-A is notoriously increased. The leakage area of the macula area is in direct proportion to the content. It indicates that the content of VEGF-A in the vitreous humor may be positively correlated with the degree of macular edema correlation. The permeability of retinal blood vessels in sufferers with macular edema reduces vascular leakage, which is beneficial to the regression of macular edema and enhances the vision of sufferers [18, 19]. Due to the complex pathogenesis and pathological changes of diabetic macular edema, anti-VEGF drug therapy has its limitations and cannot act on various pathogenic factors of DR. It is difficult to achieve the best results. The therapy effect of 1 month/time is more extensive, which can delay or reduce the development of retinal nonperfusion areas to the greatest extent [20, 21]. Anti-VEGF therapy drugs have a short half-life, and retinal neovascularization may recur after a certain period of drug metabolism. Thus, the therapy needs to be repeated within a certain period of time [22, 23].

The article "Study on BCVA, CMT, CME, Curative Effect, and Prognostic Value of DR Sufferers Based on Surgical Therapy Combined with VEGF Therapy at Different Times" was retracted in 2023. Reasons: signs of a paper mill; suspected computer-generated content; unreliable results or conclusions; concerns about the data.

## 3. Examination Objects and Methods

### 3.1. Examination Objects

In this study, DR sufferers who are treated in our hospital from March 2019 to March 2021 are selected as the examination objects. A total of 170 sufferers with 170 eyes, aged 37 to 82 years old, are randomly divided into contrast sets (85 sufferers with 85 eyes). The study set included 85 sufferers with 85 eyes. This study is approved by the Ethics Committee of our hospital, and the enrolled subjects are informed about the study and signed the informed consent.

Inclusion criteria are as follows: (1) meet the diagnostic criteria of DR; Type II diabetic sufferers with a good general condition; (2) the ocular lesions are examined by optical coherence tomography (OCT), fundus fluorescein angiography (FFA), and diagnosed with DME; and (3) before therapy, the best corrected vision (BCVA) is 0.1–0.4, and the central macular thickness (CMT) is greater than 250 *μ*m.

Exclusion criteria are as follows: (1) past history of ocular surgery, trauma, retinal detachment, glaucoma, and other ocular diseases; (2) those with poor therapy compliance or loss to follow-up; (3) intolerance or unsatisfactory effect of the therapy plan designed in this trial requires other therapy measures; (4) those who are seriously ill and need emergency therapy; (5) those with serious complications; (6) those who have used contraindicated drugs; and (7) those with missing data on cases and related impact examinations.

### 3.2. Methods

#### 3.2.1. Preoperative Examination

The visual acuity of the two sets of sufferers is detected by the international visual chart before operation. The best corrected visual acuity is obtained by optometry, and the intraocular pressure is detected by the Goldmann applanation tonometer [24]. The sufferer is in a sitting position, and the fovea is the center under the center of the macular fixation [25, 26]. The horizontal and vertical orientations of the fovea are scanned by the fast scanning method, and the CMT and SFCT are measured, recorded, and analyzed by using the OCT software. All sufferers are given levofloxacin eye drops before the operation, 4 times a day for 3 consecutive days.

#### 3.2.2. Intravitreal Injection Surgery

Intraocular pressure measurement and fundus examination are performed again on the same day to ensure the safety of the operation. After entering the operating room, the patient will be asked again if there is any discomfort. In addition, patients will be informed of matters needing attention during the operation. The operator waits for the sufferer to brake before continuing the operation. The sufferers are in a supine position, routine ophthalmic disinfection and drape, topical anesthesia with proparacaine hydrochloride eye drops, routine sterilization and drape according to the requirements of internal eye surgery, eyelid opening with eyelid opener, both sets of sufferers are extracted with 1 mL syringe Conbercept (0.05 mL/0.5 mg), inject the needle vertically at the lower temporal point 4 mm away from the corneal limbus, inject Conbercept into the vitreous cavity, slowly pull out the needle after the injection, and press the puncture point with a cotton swab to prevent a recurrence. Both sets are treated for 3 months, the contrast set is treated for 2 times, the study set is treated for 1 time/month, and the therapy frequency is 3 times. Within 3 days after therapy, the two sets of sufferers are treated with tobramycin and dexamethasone drops Eye drops, 4–6 times a day for 3 days. All operations are performed by the same physician.

The article "Study on BCVA, CMT, CME, Curative Effect, and Prognostic Value of DR Sufferers Based on Surgical Therapy Combined with VEGF Therapy at Different Times" was retracted in 2023. Reasons: signs of a paper mill; suspected computer-generated content; unreliable results or conclusions; concerns about the data.

#### 3.2.3. Observation Indicators

The observation indicators are as follows: (1) collect BCVA before therapy and 1 month, 3 months, and 6 months after therapy in the two sets, and use the international standard vision chart for BCVA examination; (2) IOP is measured by Goldmann tonometer before and after therapy; CMT and CME are measured by Cirrus HD-OCT (Zeiss, Germany) before and after therapy; (3) OCT is used to measure the total volume of neurepithelium with a diameter of 6 mm in the foveal retinal neuromacular region; (4) Image *J* software is used to calculate the vessel density (VD) of retinal capillaries before and after therapy; (5) using computer images to analyze the area of the nonperfusion area before and after therapy in the two sets; (6) statistics on the occurrence of postoperative complications in the two sets of sufferers; and (7) the cumulative recurrence within 6 months after surgery is a contrast between the two sets.

#### 3.2.4. Statistical Methods

This study collects and organizes data, establishes a corresponding database for it, and enters all the databases into SPSS 26.0 for data processing, in which the measurement data is tested for normality, expressed as (*x* ± *s*), which is consistent with the normal multi-set test as F. MANOVA spherical decomposition is used for repeated measures. The independent samples *t*-test is used for data between sets, paired samples *t*-test is used for data within sets, and Mann–Whitney *U* test is used for non-normality. When *P* < 0.05, the disparity between the data is considered to be statistically extensive.

The article "Study on BCVA, CMT, CME, Curative Effect, and Prognostic Value of DR Sufferers Based on Surgical Therapy Combined with VEGF Therapy at Different Times" was retracted in 2023. Reasons: signs of a paper mill; suspected computer-generated content; unreliable results or conclusions; concerns about the data.

## 4. Comparative Results

### 4.1. Contrast of BCVA Disparities between the Two Sets before and after Therapy

Before therapy, there is no extensive disparity in BCVA between the two sets (*P* > 0.05). After therapy, the BCVA of the two sets of sufferers is notoriously enhanced in contrast with before therapy, and the disparity is statistically extensive (*P* < 0.05). After one month, the visual acuity of BCVA is notoriously enhanced in contrast with the contrast set, and the disparity is statistically extensive (*P* < 0.05), as shown in Table 1.

### 4.2. Contrast of Disparities in CMT and CME between the Two Sets before and after Therapy

Before therapy, there is no extensive disparity in CMT and CME between the two sets (*P* > 0.05). After therapy, CMT and CME in the two sets are notoriously lower than those before therapy, and the disparity is statistically extensive (*P* < 0.05). After 3 months, the thickness of CMT and CME decreased to a higher degree than that of the contrast set (*P* < 0.05), as shown in Table 2 and Figure 1. The symbol “*∗*” indicates that contrast with before therapy, *P* < 0.05, the disparity is statistically extensive.

### 4.3. Contrast of the Total Volume of the 6 mm Diameter Neurepithelium in the Macular Region

Before therapy, there is no extensive disparity in the total macular volume of the two sets of sufferers. With the prolongation of therapy time, the overall volume of the 6 mm diameter neurepithelium in the macular area of the two sets of sufferers gradually decreased. The volume decreased more notoriously, and the disparity is statistically extensive (*P* < 0.05). The contrast between the same sets showed that the overall volume of the 6 mm diameter neurepithelium in the macular area after therapy is enhanced contrast with before therapy, and the disparities are statistically extensive (all *P* < 0.05), as shown in Table 3.  Figure 2 shows the contrast of the total volume of the 6 mm diameter neuroepithelial in the macular area before and after therapy between the two sets of sufferers.

### 4.4. Contrast of Blood Vessel Density of Retinal Capillaries before and after Therapy in the Two Sets of Sufferers

Before therapy, there is no extensive disparity in blood vessel density between the two sets. After therapy, the effect of improving the blood vessel density of retinal capillaries in the contrast set and the study set is extensive, and the disparity is statistically extensive (*P* < 0.05). The blood vessel density of retinal capillaries before and after is not notoriously enhanced, and the disparity is not statistically extensive (all *P* < 0.05), as shown in Table 4 and Figure 3.

The article "Study on BCVA, CMT, CME, Curative Effect, and Prognostic Value of DR Sufferers Based on Surgical Therapy Combined with VEGF Therapy at Different Times" was retracted in 2023. Reasons: signs of a paper mill; suspected computer-generated content; unreliable results or conclusions; concerns about the data.

### 4.5. Contrast of the Area of the Central Nonperfusion Area before and after Therapy between the Two Sets of Sufferers

Before therapy, there is no extensive disparity in the area of the central nonperfusion area between the two sets of sufferers. After therapy, the area of the central nonperfusion area in the two sets is enhanced. By comparison to the contrast set, the enhancement in the area of the central nonperfusion area in the study set is more extensive, and the disparity is statistically extensive (*P* < 0.05). The contrast between the same sets showed that the area of the central nonperfusion area after therapy is enhanced contrast with before therapy, and the disparity is statistically extensive (all *P* < 0.05), as shown in Table 5 and Figure 4.

### 4.6. Contrast of Adverse Reactions between the Two Sets of Sufferers after Therapy

There is no extensive disparity in the incidence of adverse reactions between the two sets after therapy (all *P* > 0.05). Both sets had the highest incidence of the mild subconjunctival hemorrhage, and no serious complications such as endophthalmitis and retinal detachment occurred, as shown in Table 6.

### 4.7. Cumulative Recurrence Rate within 6 Months after Therapy in the Two Sets

Both sets are followed up for 6 months. During the follow-up period, the recurrence rate of the study set is 7.06%, which is notoriously lower than that of the contrast set. The disparity is statistically extensive (*P* < 0.05), as shown in Figure 5.

## 5. Conclusions

In this study, the efficacy and prognostic value of BCVA, CMT, and CME in DR sufferers based on surgical therapy combined with VEGF therapy at different times are investigated. The BCVA, CMT, and CME of the two sets before and after therapy are observed. The 6 mm diameter neuroepithelial volume, retinal capillary VD and the area of the nonperfusion area in the macular fovea retinal neuromacular area before and after therapy are observed in the two sets. The incidence of related complications and the cumulative recurrence within 6 months after surgery are compared between the two sets. The BCVA of the two sets was notoriously enhanced. The visual acuity of the study set is notoriously enhanced in contrast with the contrast set; the CMT and CME of the two sets are notoriously lower than those before therapy. CMT and CME in the study set decreased more than those in the contrast set. The blood vessel density of retinal capillaries in the contrast set and the examination set was notoriously enhanced. Although this study achieves certain examination results, only 6 months of follow-up is performed on the sufferers, and the long-term efficacy cannot be determined. In future work, the follow-up time should be further increased to analyze the clinical effects of anti-VEGF therapy in DR sufferers at different times.

The article "Study on BCVA, CMT, CME, Curative Effect, and Prognostic Value of DR Sufferers Based on Surgical Therapy Combined with VEGF Therapy at Different Times" was retracted in 2023. Reasons: signs of a paper mill; suspected computer-generated content; unreliable results or conclusions; concerns about the data.

## Figures and Tables

**Figure 1:** Contrast of CMT before and after therapy in the two sets of sufferers.

**Figure 2:** Contrast of the total volume of the 6 mm diameter neuroepithelial in the macular area before and after therapy between the two sets of sufferers.

**Figure 3:** Contrast of the blood vessel density of retinal capillaries before and after therapy in the two sets of sufferers.

**Figure 4:** Contrast of the area of the central nonperfusion area before and after therapy in the two sets of sufferers.

**Figure 5:** The cumulative recurrence rate curve within 6 months after therapy in the two sets of sufferers.

**Table 1:** Contrast of BCVA disparities between the two sets of sufferers before and after therapy.

Set	Number of cases	Before therapy	1-month therapy	3-month therapy
Examination set	85	1.63 ± 0.13	0.56 ± 0.13	0.43 ± 0.16
Contrast set	85	1.61 ± 0.19	0.76 ± 0.14	0.61 ± 0.05
*t*		5.263	2.639	6.371
*P*		0.737	0.001	<0.001

**Table 2:** Contrast of disparities in CMT and CME between the two sets before and after therapy.

Set	Number of cases	CMT		CME	
		Before therapy	3-month therapy	Before therapy	3-month therapy
Examination set	85	521.11 ± 116.1	204.46 ± 110.4 ^*∗*^	1115.23 ± 213.52	0.00 ± 0.00 ^*∗*^
Contrast set	85	522.66 ± 120.1	250.44 ± 100.1 ^*∗*^	1126.38 ± 225.49	233.25 ± 156.63 ^*∗*^
*t*		0.296	3.771	0.395	23.529
*P*		0.877	0.001	0.791	0.001

**Table 3:** Contrast of the total volume of the 6 mm diameter neurepithelium in the macular area before and after therapy in the two sets of sufferers.

Set	Number of cases	Before therapy	1-month therapy	3-month therapy
Examination set	85	21.53 ± 4.27	13.81 ± 2.17 ^*∗*^	8.52 ± 2.12 ^*∗*^
Contrast set	85	21.08 ± 4.29	16.89 ± 3.15 ^*∗*^	12.57 ± 2.13 ^*∗*^
*t*		0.632	3.625	7.526
*P*		0.528	0.001	0.001

**Table 4:** Contrast of blood vessel density of retinal capillaries before and after therapy in two sets of sufferers (*x* ®± *s*).

Set	Number of cases	Before therapy	1-month therapy	3-month therapy
Examination set	85	44.53 ± 0.27	42.82 ± 0.04 ^*∗*^	42.12 ± 0.14 ^*∗*^
Contrast set	85	44.48 ± 0.29	43.83 ± 0.03 ^*∗*^	43.57 ± 0.21 ^*∗*^
*t*		0.532	4.362	8.153
*P*		0.617	0.001	0.001

**Table 5:** Contrast of the area of the central nonperfusion area before and after therapy in the two sets of sufferers (*x* ®± *s*).

Set	Number of cases	Before therapy	1-month therapy	3-month therapy
Examination set	85	1.83 ± 4.22	1.64 ± 0.32 ^*∗*^	1.57 ± 0.15 ^*∗*^
Contrast set	85	1.88 ± 3.28	1.82 ± 0.11 ^*∗*^	1.75 ± 0.11 ^*∗*^
*t*		0.532	4.362	8.153
*P*		0.617	0.001	0.001

The article "Study on BCVA, CMT, CME, Curative Effect, and Prognostic Value of DR Sufferers Based on Surgical Therapy Combined with VEGF Therapy at Different Times" was retracted in 2023. Reasons: signs of a paper mill; suspected computer-generated content; unreliable results or conclusions; concerns about the data.

**Table 6:** Complications after therapy in two sets of sufferers [*n* (%)].

Set	Number of cases	Mild subconjunctival hemorrhage	Endophthalmitis	Pigment epithelial damage	Retinal detachment	Total
Examination set	85	3	0	2	0	5 (5.88)
Contrast set	85	3	0	3	0	6 (7.06)
*χ* ^2^						0.632
*P*						0.518

## Data Availability

The simulation experiment data used to support the findings of this study are available from the corresponding author upon request.
